The article "Epithelial Mesenchymal Transition Is Required for Acquisition of Anoikis Resistance and Metastatic Potential in Adenoid Cystic Carcinoma" was retracted in 2014. Reasons: errors in the cell lines or tissues; unreliable results or conclusions.

# Epithelial Mesenchymal Transition Is Required for Acquisition of Anoikis Resistance and Metastatic Potential in Adenoid Cystic Carcinoma

**DOI:** 10.1371/journal.pone.0051549

**Published:** 2012-12-14

**Authors:** Jun Jia, Wei Zhang, Jian-Ying Liu, Gang Chen, Hui Liu, Hao-Yan Zhong, Bing Liu, Yu Cai, Jia-Li Zhang, Yi-Fang Zhao

**Affiliations:** 1 The State Key Laboratory Breeding Base of Basic Science of Stomatology and Key Laboratory of Oral Biomedicine Ministry of Education, School and Hospital of Stomatology, Wuhan University, Wuhan, China; 2 Department of Oral and Maxillofacial Surgery, School and Hospital of Stomatology, Wuhan University, Wuhan, China; 3 Department of Pathology, School and Hospital of Stomatology, Wuhan University, Wuhan, China; University Magna Graecia, Italy

## Abstract

Human adenoid cystic carcinoma (ACC) is characterized by diffused invasion of the tumor into adjacent organs and early distant metastasis. Anoikis resistance and epithelial mesenchymal transition (EMT) are considered prerequisites for cancer cells to metastasize. Exploring the relationship between these processes and their underlying mechanism of action is a promising way to better understand ACC tumors. We initially established anoikis-resistant sublines of ACC cells; the variant cells revealed a mesenchymal phenotype through Slug-mediated EMT-like transformation and displayed enhanced metastatic potential both *in vitro* and *in vivo*. Suppression of EMT by knockdown of Slug significantly impaired anoikis resistance, migration, and invasion of the variant cells. With overexpression of Slug and Twist, we determined that induction of EMT in normal ACC cells could prevent anoikis, albeit partially. These findings strongly suggest that EMT is indispensable in anoikis resistance, at least in ACC cells. Furthermore, we found that the EGFR/PI3K/Akt pathway acts as the common regulator for EMT-like transformation and anoikis resistance, as confirmed by their specific inhibitors. Gefitinib and LY294003 restored the sensibilities of anoikis-resistant cells to anoikis and simultaneously impaired their metastatic potential. In addition, the results from our *in vivo* model of metastasis suggest that pretreatment with gefitinib promotes mouse survival by alleviating pulmonary metastasis. Most importantly, immunohistochemistry of human ACC specimens showed a correlation between the overexpression of Slug and EGFR staining. This study has demonstrated that Slug-mediated EMT-like transformation is required by human ACC cells to achieve anoikis resistance and their metastatic potential. Targeting the EGFR/PI3K/Akt pathway holds potential as a preventive strategy against distant metastasis of ACC.

The article "Epithelial Mesenchymal Transition Is Required for Acquisition of Anoikis Resistance and Metastatic Potential in Adenoid Cystic Carcinoma" was retracted in 2014. Reasons: errors in the cell lines or tissues; unreliable results or conclusions.

## Introduction

Adenoid cystic carcinoma (ACC) is one of the most common malignancies of the major and minor salivary glands [1] that accounts for approximately 15%–25% of all malignant salivary gland carcinomas [1], [2]. Typically, ACC grows slowly, but it spreads relentlessly into adjacent tissues and develops distant metastasis frequently to the lungs, bone, and soft tissues. Most patients with ACC (80%–90%) die within 10–15 years after being diagnosed due to high rates of recurrence and distant metastasis [3]. Although numerous studies have identified the factors related to the prognosis and outcome of ACC, little is known about the underlying molecular mechanisms that control its ability to spread to distant organs. A better understanding of the biological process involved in ACC metastasis is therefore urgently needed.

Metastasis is a multistep process in which cancer cells spread from the primary site to distant organs through the lymphatic or circulatory system [4], [5]. In normal epithelial cells, loss of cell–cell or cell–matrix interactions triggers a form of apoptosis known as anoikis, which inhibits the survival of cancer cells in the circulation [6]. Thus, their survivability in anchorage-independent environments, such as dissemination in the circulatory system, is considered a prerequisite for cancer cells to metastasize. Epithelial mesenchymal transition (EMT) describes a series of rapid changes in the cellular phenotype in which epithelial cells down-modulate their adhesion structures, alter their polarity, and adopt a mesenchymal morphology [7]. EMT is essential for the formation of mesodermal tissue from early embryonic epithelial cells during development, and it is associated with wound healing, tissue inflammation, and organ fibrosis in adults [7], [8]. Accumulating evidence suggests that an EMT-like transformation contributes to tumor progression in most cases, including human ACC [9], [10]. Recent studies have shown that transformation not only endows cancer cells with motility to detach from neighboring cells but also promotes anoikis resistance in cancer cells in anchorage-independent circumstances [11], [12]. The crosstalk between integrin–extracellular matrix (ECM) and growth factors involved in EMT also exists between the pathways related to anoikis resistance [13], [14]. More recent studies have demonstrated that cancer cells undergo an EMT-like transformation in the peripheral circulation of patients with carcinomas [15]–[17], strongly suggesting that EMT contributes to anoikis resistance. Exploring the relationship between anoikis resistance and EMT and their common mechanism of action is thus a promising way of better understanding metastasis.

The article "Epithelial Mesenchymal Transition Is Required for Acquisition of Anoikis Resistance and Metastatic Potential in Adenoid Cystic Carcinoma" was retracted in 2014. Reasons: errors in the cell lines or tissues; unreliable results or conclusions.

In this study, we established anoikis-resistant variants of ACC cells to investigate the involvement of EMT-like transformation in the acquisition of anoikis resistance. We found that Slug-mediated EMT promotes cell motility and contributes to the acquisition of anoikis resistance. We also found that activation of the epidermal growth factor receptor (EGFR, ErbB-1, HER1)/phosphoinositide-3 kinase (PI3K)/Protein Kinase B (PKB, Akt) signaling pathway is the common mechanism of EMT and anoikis resistance in activated ACC cells. Using a pharmacological inhibitor of EGFR, we succeeded in delaying pulmonary metastasis in nude mice injected with these variant cells and promoting their survival, which suggests that targeting the EGFR/PI3K/Akt pathway holds potential in preventing metastasis of human ACC.

## Materials and Methods

### Chemicals and Antibodies

Poly(2-hydroxyethyl methacrylate) [poly(HEMA)], dimethyl sulfoxide (DMSO), Hoechst 33258, LY294002, and G418 were purchased from Sigma-Aldrich (St. Louis, MO, USA). Gefitinib was purchased from Selleck Chemicals (Houston, TX, USA). Dulbecco’s modified Eagle’s medium (DMEM), fetal bovine serum (FBS), penicillin, and streptomycin were obtained from GIBCO (Carlsbad, CA, USA). Primary antibodies against human phospho-EGFR (Tyr1068), phospho-PI3K p85 (Tyr458), phospho-Akt (Ser473), Slug, cleaved caspase-3, cleaved caspase-9, and cleaved poly(ADP-ribose) polymerase (PARP) were purchased from Cell Signaling Technology (Danvers, MA). Primary antibodies against PI3K p85, Akt, Bax, Bcl-2, EGF, matrix metalloproteinase 9 (MMP9), and actin were purchased from Santa Cruz Biotechnology, Inc. (Santa Cruz, CA). Primary antibodies against E-cadherin, N-cadherin, α-smooth muscle actin, vimentin, and Twist were purchased from Epitomics, Inc. (Burlingame, CA, USA). Recombinant EGF was purchased from Cell Signaling Technology as well.

### Cell Culture and Generation of Anoikis-Resistant Variants

The high (ACC-M) and low (ACC-2) metastatic cell lines of human salivary ACC were obtained from the China Center for Type Culture Collection [18] and maintained in DMEM supplemented with 10% FBS (v/v), 100 U/ml penicillin, and 100 mg/ml streptomycin. The cells were incubated in a humidified atmosphere of 95% air and 5% CO_2_ at 37°C.

Poly(HEMA) was prepared by dissolving it in 95% ethanol (v/v) to a concentration of 20 mg/ml and subsequently added to cell culture wells at a density of 5 mg/cm^2^. The dishes were then allowed to dry overnight. Anoikis-resistant ACC cells (ACC^Ar^) were generated by sequential cycles of culture using poly(HEMA)-treated (suspended) and untreated (adhered) dishes. Briefly, ACC monolayers were trypsinized, transferred to poly(HEMA)-treated dishes for 3 days of culture and then to untreated dishes, and allowed to replicate for 1 day. The variants were harvested after six rounds of culture and then labeled as ACC^Ar^ cells.

The article "Epithelial Mesenchymal Transition Is Required for Acquisition of Anoikis Resistance and Metastatic Potential in Adenoid Cystic Carcinoma" was retracted in 2014. Reasons: errors in the cell lines or tissues; unreliable results or conclusions.

### Clinical Samples and Immunohistochemistry

Fifty pathologically confirmed human ACC specimens with six corresponding pericancerous normal salivary gland tissues were collected at the Hospital of Stomatology, Wuhan University. All specimens were fixed in 4% buffered paraformaldehyde and embedded in paraffin. The procedures were performed in accordance with the National Institutes of Health guidelines for the use of human tissues. The study was approved by the review board of the Ethics Committee of the Wuhan University Hospital of Stomatology. Written informed consent was obtained from all study participants. Immunohistochemical analysis was performed according to our previous procedures [18], as described in Protocol S1.

### Transfection and Infection with Lentivirus

pEGFP-N1-SNAI2-GFP (pEGFP-Slug) and pEGFP-N1-TWIST1-GFP (pEGFP-Twist) were purchased from Genechem (Shanghai, China). The constructs were confirmed to be correct by restriction enzyme digestion and sequencing. The stably transfected ACC-2 cell lines of pEGFP-Twist and pEGFP-Slug were selected by G418 (500 µg/ml) for 2 weeks and confirmed by reverse transcription (RT)-PCR and Western blot analysis. For siRNA-mediated inhibition, three siRNA sequences against human Slug (5′-AACTGGACACACATACAGTG-3′, 5′-CAGACCCATTCTGATGTAAAG-3′, and 5′-GAGGAAAGACTACAGTCCAAG-3′) were cloned into pBRsi-hU6 lentiviral vector systems (Slug siRNA 1, Slug siRNA 2, and Slug siRNA 3). The negative control (NC) siRNA and lentiviral vector package were provided by Genechem. The RNA interference (RNAi) efficiency of the three constructs was confirmed by RT-PCR and Western blot analysis. According to the results, Slug siRNA 2 was selected for the formal experiments (Figure S3).

### Cell Growth Analysis and Viability Measurement

MTT assay was performed to measure the growth curves of ACC and ACC^Ar^ cells. Briefly, 2000 cells/well were plated onto 96-well plates and incubated for 24, 48, and 72 h with 100 µl of DMEM. Then, 10 µl of MTT (5 mg/ml) was added to each well, which was incubated for another 4 h. Afterwards, the supernatant was discarded with 100 µl of dimethyl sulfoxide added to each well. Absorbance was assessed at 490 nm using a 96-well microplate reader (Bio-Tek). Cell viability was measured with a Vi-CELL Cell Viability Analyzer (Beckman Coulter, Fullerton, CA) based on trypan blue exclusion (TBE) assays.

### Determination of Apoptosis

Apoptosis induction by the detachment in ACC or ACC^Ar^ cells was determined according to our previous procedures [18] as follows: (a) morphological evaluation by Hoechst staining; (b) quantitation of cytoplasmic histone-associated DNA fragments with Cell Death Detection ELISA^PLUS^; and (c) Western blot analysis for Bax/Bcl-2 ratio, caspase-3, caspase-9, and PARP cleavage.

The article "Epithelial Mesenchymal Transition Is Required for Acquisition of Anoikis Resistance and Metastatic Potential in Adenoid Cystic Carcinoma" was retracted in 2014. Reasons: errors in the cell lines or tissues; unreliable results or conclusions.

### Wound Healing Assay

ACC and ACC^Ar^ cells were seeded in six-well culture plates (Corning Life Sciences, NY) and allowed to grow to 90% confluence. The center of the cell monolayers was scraped with a sterile micropipette tip to create a gap of constant width. After 12 h, the cells that migrated into the gap were counted after fixation and observed under a phase microscope (Leica).

### Migration and Invasion Assays

The ability of ACC and ACC^Ar^ cells to pass through filters was measured using a transwell Boyden chamber system (Corning Life Sciences) containing a polycarbonate filter (6.5 mm diameter; pore size of 8 µm). Matrigel was diluted to 200 µg/ml and applied to the top side of the filter in the cell invasion assay. In contrast, the filter was not coated in the cell migration assay. ACC and ACC^Ar^ cells were seeded in the upper chamber at a density of 10^4^ cells/well in 100 µl of serum-deprived medium, whereas 10% FBS medium was applied to the lower chamber as chemoattractant. After incubation for 24 h at 37°C, the cells in the upper surface of the membrane were carefully removed with a cotton swab, and migrated cells were fixed with methanol, stained with eosin, and then photographed and quantified.

### Soft Agar Assay

For soft agar assay, 2000 trypsinized cells were seeded in 0.4% low-melting-point agarose (Takara, Kyoto, Japan) on top of a 1% agarose layer, and scans were taken 11 days later. The number of macroscopic colonies was determined using ImageJ software (http://rsb.info.nih.gov/ij/index.html).

### Immunofluorescence Analysis for Cells

The localization of E-cadherin and Vimentin was detected by indirect immunofluorescence analysis. In brief, ACC cells were grown on glass coverslips with indicated treatment. Then, cells were washed with PBS, fixed in 100% methanol at −20°C, and blocked in 10% non-immune goat serum for 1 h at room temperature. Then cells were incubated with indicated primary antibody with dilution of 1∶200 overnight at 4°C followed by incubation with Dylight488-conjugated goat anti-mouse IgG (1∶400, Jackson, West Grove, PA) for 1 h at room temperature. The nuclei were stained with DAPI and the coverslips were mounted on a microscope slide with embedding medium. The cells were observed and photographed with a fluorescence microscope (Leica).

The article "Epithelial Mesenchymal Transition Is Required for Acquisition of Anoikis Resistance and Metastatic Potential in Adenoid Cystic Carcinoma" was retracted in 2014. Reasons: errors in the cell lines or tissues; unreliable results or conclusions.

### Quantitative Real-Time RT-PCR

Quantitative real-time RT-PCR was performed to evaluate the mRNA expression levels of EMT-related genes, growth factors, and MMPs of the ACC^Ar^ cells. Total RNA was isolated with TRIzol Reagent (Invitrogen). Aliquots (1 µg) of RNA were reverse transcribed to cDNA (20 µl) with oligo(dT) and M-MuLV reverse transcriptase (Fermentas, Glen Burnie, MD). One-fifth of the cDNA was used as a template for PCR using SYBR Premix Ex Taq™ (Perfect Real Time) kits (Takara, Kyoto, Japan) in an ABI 7500 Real-Time PCR System (Applied Biosystems, Foster City, CA). 18s rRNA was selected as an internal control for each experiment. See Protocol S1 for the primer sequences designed for PCR.

### Western Blot Analysis

The proteins in corresponding cells were collected, and the concentration of protein in supernatants was estimated using BCA assay (Pierce Chemical, Rockford, IL). Subsequently, 40 mg of protein was separated on 10% SDS-polyacrylamide gels and electroblotted on polyvinylidene fluoride membranes (Roche Applied Science, Germany). The blots were blocked overnight with 5% nonfat dry milk and probed with primary antibodies at dilutions recommended by the suppliers. Immunoblots were detected by horseradish peroxidase-conjugated secondary antibody (Pierce) using a chemiluminescence kit (Pierce) and photographed.

### Mouse Model of Pulmonary Metastasis

Female BALB/c nude mice (18–20 g; 6–8 weeks old) were purchased from the Center for Animal Experiment of Wuhan University in pressurized ventilated cages according to institutional regulations. All studies were approved and overseen by the Institutional Animal Care and Use Committee, Center for Animal Experiment, Wuhan University. ACC-2, ACC-2 pretreated with EGF (10 ng/ml) for 1 h, ACC-2^Ar^, and ACC-2^Ar^ cells pretreated with gefitinib (1 µM) for 1 h (2×10^6^ in 0.1 ml of PBS) were collected from subconfluent culture and inoculated intravenously into the caudal vein of the mice. Mice were inspected daily and euthanized by CO_2_ when clinical symptoms became apparent. Lung tissues were exteriorized carefully, fixed in 4% buffered paraformaldehyde, and embedded in paraffin. Metastatic lesions in the lungs were counted by visual inspection of hematoxylin and eosin-stained histological tissue sections. The sizes of metastases and the area of lung tissue per section were determined with ImageJ software.

### Statistical Analysis

All values were expressed as the mean ± SE of three independent experiments. Data analyses were conducted using OriginPro 8.6.0 (OriginLab Corporation, Northampton, MA). Image analyses for soft agar assays were conducted using ImageJ software (http://rsb.info.nih.gov/ij/index.html). One-way ANOVA, the Student–Newman–Keuls test, and Spearman’s rank correlation test were used for statistical analysis. *p*<0.05 was considered statistically significant.

The article "Epithelial Mesenchymal Transition Is Required for Acquisition of Anoikis Resistance and Metastatic Potential in Adenoid Cystic Carcinoma" was retracted in 2014. Reasons: errors in the cell lines or tissues; unreliable results or conclusions.

## Results

### Establishment of Anoikis-Resistant Sublines of ACC Cells

Dishes treated with poly(HEMA) were used to induce anoikis-resistant sublines in both ACC cell lines. ACC-2^Ar^ and ACC-M^Ar^, referred to as the anoikis-resistant sublines of ACC-2 and ACC-M cells, respectively, were established after six alternating cycles of culture under suspension and adhesion (Figure 1A). Cells were inoculated in the dishes coated with poly(HEMA) to identify whether the variants could escape the apoptosis induced by detachment. TBE assay showed that the cell viabilities of anoikis-resistant variants were much higher than those of parental cells (Figure 1B). After culture in suspension for 24 h, several apoptotic morphological features, such as apoptotic bodies, cell shrinkage, and chromatin condensation, were observed in normal ACC cells, but they were not detected in ACC^Ar^ cells (Figure 1C). Quantitative assessment using Cell Death Detection ELISA^PLUS^ showed that the anoikis fractions of ACC-2^Ar^ and ACC-M^Ar^ cells were 0.887 and 0.501, respectively, compared with 0.256 and 0.170 in the parental cells (*p*<0.05) (Figure 1D). The results of anchorage-independent growth assay in soft agar indicated that ACC^Ar^ cells acquired the ability to survive in an anchorage-independent environment (Figure 1E). The cleavage of caspase-3, caspase-8, caspase-9, and poly (ADP-ribose) polymerase (PARP) as well as the expression of Bcl-2 and Bax were subjected to Western blot analysis to further investigate the mechanism underlying cell death. As shown in Figure 1F, the cleavage of capase-3 and that of caspase-9 were significantly augmented in normal ACC cells; however, cleavage of caspase-8 was not detected (data not shown), indicating that detachment induced anoikis via an intracellular apoptotic pathway. In addition, the Bcl-2/Bax ratio was diminished in normal ACC cells. In summary, the ACC cells cultured in suspension conditions for several rounds succeeded in acquisition the characteristic of anoikis resistance.

**Figure 1:** Establishment of anoikis-resistant sublines of ACC cells. A, Schematic of establishing anoikis-resistant sublines of ACC by cycles of culture under suspension and adhesion. B, The cell viabilities of ACC and ACC^Ar^ in suspension were measured using TBE assay (Mean ± SE, **p<0.01 versus ACC-2, ^##^ *p*<0.01 versus ACC-M). C, Hoechst 33258 staining was performed to detect the apoptosis of ACC and ACC^Ar^ cells that cultured in suspension. D, DNA fragments of ACC and ACC^Ar^ in suspension were detected using Cell Death Detection ELISA^PLUS^ (Mean ± SE, **p<0.01 versus ACC-2, ^##^ *p*<0.01 versus ACC-M). E, Anchorage-independent growth of ACC and ACC^Ar^ cells was analyzed using soft agar assay. F, Expression levels of cleaved PARP, cleaved caspase-3, cleaved caspase-9, Bax, and Bcl-2 were determined using Western blot analysis (**p<0.01 versus ACC-2, ^##^ *p*<0.01 versus ACC-M).

The article "Epithelial Mesenchymal Transition Is Required for Acquisition of Anoikis Resistance and Metastatic Potential in Adenoid Cystic Carcinoma" was retracted in 2014. Reasons: errors in the cell lines or tissues; unreliable results or conclusions.

### Anoikis-Resistant Sublines of ACC are more Aggressive in Metastasis *In Vitro*

As the acquisition of anoikis resistance is generally correlated with increased ability of migration and invasion in the progression of tumors, we measured the migration and invasion of ACC cells using wound healing and transwell Boyden chamber assays. ACC-2^Ar^ and ACC-M^Ar^ both showed enhanced migration and invasion compared with normal ACC cells (Figure 2A–D). The effects of cell proliferation on migration were excluded because the proliferation curve of ACC^Ar^ cells showed an even lower proliferation rate in both the ACC-2 and ACC-M variants (Figure S1). Our results revealed that the mRNA expression levels of vascular endothelial growth factor (VEGF), matrix metallopeptidase 9 (MMP9), and stromal cell-derived factor-1 alpha (SDF-1α) were up-regulated in ACC cells as they gained anoikis resistance (Figure 2E), which can account for the increased migration and invasion abilities of the variant cell lines. Taken together, these results revealed that the ACC^Ar^ cells selected by suspended culture displayed much more aggressive potential than their parental cells both *in vitro*.

**Figure 2:** Enhanced migration and invasion of ACC^Ar^ cells. A and B, The migration of ACC and ACC^Ar^ was analyzed using wound healing and transwell Boyden system assays. C, The invasion of ACC and ACC^Ar^ was measured using a transwell Boyden system coated with Matrigel. D, Quantification of migrated and invaded cells in wound healing assays and transwell migration/invasion assays. The results were represented as relative ratio to ACC-2 (Mean ± SE, **p<0.01 versus ACC-2, ^##^ *p*<0.01 versus ACC-M). E, The relative mRNA expression levels of VEGF, MMP9, and SDF-1α were analyzed by real-time RT-PCR. The results were represented as relative ratio to ACC-2 (Mean ± SE, **p<0.01 versus ACC-2, ^##^ *p*<0.01 versus ACC-M).

### ACC^Ar^ Cells Undergo EMT-Like Transformation in Attachment Culture

Simultaneous with the detection of the migration and invasion abilities of ACC^Ar^ cells, their morphological transformation from cobblestones to an elongated, spindle-shaped appearance was observed (Figure 3A). As the acquisition of anoikis resistance is widely considered to generally be accompanied by morphological EMT-like changes, we decided to further verify the nature of this transformation. As shown in Figure 3A, E-cadherin was correctly localized at the adherent junctions in normal ACC cells, but they were lost in the ACC^Ar^ cells. Simultaneously, vimentin as a mesenchymal marker notably increased in ACC-2^Ar^ cells, compared with its negative expression in ACC-2 cells (Figure 3A). Moreover, the results from western blots and qPCR showed the expression levels of several epithelial markers were down-regulated with the up-regulation of mesenchymal proteins at the mRNA and protein levels (Figure 3B and C, Figure S2). The expression level of vimentin in ACC-M cells was higher than that in ACC-2 cells, which might be responsible for the more aggressive nature of ACC-M cells compared with ACC-2 cells [19], [20]. However, the ACC^Ar^ cells would lose their mesenchymal features when cultured in adhesion for 6 days, indicating that EMT-like transformation might be a transient process.

The article "Epithelial Mesenchymal Transition Is Required for Acquisition of Anoikis Resistance and Metastatic Potential in Adenoid Cystic Carcinoma" was retracted in 2014. Reasons: errors in the cell lines or tissues; unreliable results or conclusions.

**Figure 3:** EMT-like transformation in ACC^Ar^ cells. A, A mesenchymal morphology as well as epithelial (E-cadherin) and mesenchymal (vimentin) markers were detected in ACC-2^Ar^ and ACC-M^Ar^. B, Protein expression levels of EMT-related genes in ACC^Ar^ cells were measured using Western blot analysis. C, The mRNA expression levels of E-cadherin, N-cadherin, and vimentin in ACC^Ar^ cells were determined using qRT-PCR. D, The mRNA expression levels of Snail, Slug, and Twist in ACC^Ar^ cells were determined using qRT-PCR. E, The mRNA expression levels of bone morphogenetic protein 4 (BMP4) and connective tissue growth factor (CTGF) in ACC^Ar^ cells were determined using qRT-PCR. The results of qRT-PCR were represented as relative ratio to ACC-2 cells (Mean ± SE, **p<0.01 versus ACC-2, ^##^ *p*<0.01 versus ACC-M).

Several transcription factors that repress epithelial genes, such as those encoding E-cadherin and cytokeratins, via E-boxes in the corresponding promoters include Twist and members of the Snail protein family. We then assessed the mRNA and protein expression levels of these transcription factors, which played critical roles in the EMT process (Figure 3B and D). Our results showed that Slug was significantly up-regulated, Twist slightly increased, and the expression level of Snail did not significantly change in ACC^Ar^ cells. In addition, we measured previously reported EMT-related cytokines, and the qPCR results revealed that the mRNA expression of connective tissue growth factor (CTGF) was up-regulated, however no change in bone morphogenetic protein 4 (BMP4) was determined (Figure 3E). In summary, our results suggest that EMT-like transformation is strongly induced by the acquisition of anoikis resistance in ACC cells. Most importantly, we found that ACC-2^Ar^ showed more prominent anoikis resistance, migration, invasion, and EMT-like transformation compared with its parental cells than the ACC-M cell line. Thus, ACC-2^Ar^ and its parental cells were chosen for further investigation.

The article "Epithelial Mesenchymal Transition Is Required for Acquisition of Anoikis Resistance and Metastatic Potential in Adenoid Cystic Carcinoma" was retracted in 2014. Reasons: errors in the cell lines or tissues; unreliable results or conclusions.

### Activation of the EGFR/PI3K/Akt Signaling Pathway Moderates the Acquisition of Anoikis Resistance and EMT-Like Transformation

Previous research has shown that growth factors, such as transforming growth factor-beta 1 (TGF-β1), epithelial growth factor (EGF), and hepatocyte growth factor (HGF), among others, induce EMT-like transformation and anoikis suppression in epithelial cells [21], [22]. Thus, we assessed those EMT inducers at the mRNA expression level. As shown in Figure 4A, EGF was strongly induced in the process of establishment of ACC^Ar^ cells, which was further confirmed by Western blot analysis. In addition, the phosphorylation level of its receptor, EGFR, was augmented simultaneously (Figure 4B). Furthermore, stimulation with EGF (10 ng/ml) for 48 h was sufficient to induce EMT-like changes in normal ACC cells, strongly suggesting the essential role of the EGFR signaling pathway in EMT induction of ACC^Ar^ cells (Figure 4C and D). Gefitinib (1 µM), a specific inhibitor for EGFR, effectively suppressed the activation of EGFR and reverted the spindle-shaped appearance of ACC-2^Ar^ cells back to their epithelial shape in adhesion (Figure 4C and D). Moreover, treatment with gefitinib negatively affected the apoptosis evasion of variants in detachment and their migration capabilities (Figure 4E and F).

**Figure 4:** Involvement of EGFR/PI3K/Akt pathway in acquisition of anoikis resistance and EMT-like transformation in ACC^Ar^ cells. A, The mRNA expression levels of EGF in ACC^Ar^ cells were measured using qRT-PCR, and results were expressed as relative ratio to ACC-2 cells (Mean ± SEM, **p<0.01 versus ACC-2, ^##^ *p*<0.01 versus ACC-M). B, The protein expression levels of EGFR, PI3K, Akt, and their phosphorylated forms in ACC and ACC^Ar^ cells were determined using Western blot analysis. C, The transformed ACC-2 cells (both ACC^Ar^ and EGF-treated cells) were treated with gefitinib (1 µM) and LY294002 (10 µM) for 12 h before detection. The parental ACC-2 cells were used as Control. The expression levels of the phosphorylated form of EGFR, Akt, and E-cadherin, vimentin, and Slug were subjected to Western blot analysis. D, A mesenchymal morphology as well as epithelial (E-cadherin) and mesenchymal (vimentin) markers were detected in ACC cells with indicated treatment as describe above. E, The apoptosis rate in suspension was analyzed using Cell Death Detection ELISA^PLUS^ (Mean ± SE, *p<0.05, **p<0.01 versus ACC-2; ^##^ *p*<0.01 versus ACC-2^Ar^). F, The migration of ACC cells with indicated treatment was analyzed using transwell Boyden system.

The article "Epithelial Mesenchymal Transition Is Required for Acquisition of Anoikis Resistance and Metastatic Potential in Adenoid Cystic Carcinoma" was retracted in 2014. Reasons: errors in the cell lines or tissues; unreliable results or conclusions.

Previous studies have demonstrated that the PI3K/Akt and mitogen-activated protein kinase (MAPK) pathways are up-regulated by EGFR activation, leading to EMT and cellular migration [10], [23], [24]. The key kinases of these signaling cascades were subjected to Western blot analysis. The results showed that the PI3K/Akt pathway was activated in the variants and that the phosphorylation status of extracellular regulated protein kinases (ERK), p38 mitogen-activated protein kinase (p38 MAPK), and c-Jun N-terminal kinase (JNK) did not change. Furthermore, several pharmacological inhibitors were used to further confirm the involvement of the corresponding signaling pathway, showing that specific inhibitors of MAPK/ERK kinase (MEK) (U0126), p38 (SB203580), and JNK (SP600125) did not affect transformation and aggression in ACC-2^Ar^ cells (data not shown). However, suppression of the PI3K/Akt signaling pathway with LY294002 (10 µM) abrogated the augmentation of Slug expression induced by EGFR activation and restored E-cadherin levels in ACC-2^Ar^ cells, accompanied by a reversal from their spindle-shaped cell morphology toward an epithelial appearance (Figure 4C and D). Moreover, inhibition of PI3K/Akt signaling inhibited enhanced migration and invasion in ACC-2^Ar^ cells (Figure 4F). Collectively, these results demonstrated that activation of EGFR induced the acquisition of anoikis resistance in ACC^Ar^ cells, led to EMT-like transformation, and enhanced metastatic potential mainly via the EGFR/PI3K/Akt signaling pathway.

### Gefitinib Suppresses the Enhanced Metastasis of Anoikis-Resistant Sublines of ACC *In Vivo*

To determine the enhanced metastatic capability of ACC^Ar^ and the preventive effects of gefitinib against the metastatic abilities of these cells *in vivo*, we injected cells with distinct pretreament (ACC-2^Ar^ was selected for the marked improvement in its migration and invasion abilities compared with ACC-M^Ar^) into nude mice intravenously to establish an *in vivo* metastasis model. Our results indicated that the ACC-2^Ar^ cells significantly shortened the life span of mice compared with normal ACC-2 cells. After the mice were sacrificed, each organ was imaged and retained. Growth of the anoikis-resistant subline cells was detected in the lung, reflecting the metastatic tendency of ACC. The incidence of metastasis was measured by the number of pulmonary metastatic clones (Figure 5A and B). Consistent with our *in vitro* studies, ACC-2^Ar^ showed much enhanced metastatic ability in the model and displayed a much shorter life span (Figure 5C and D). Most importantly, pretreatment with gefitinib suppressed the formation of metastatic lesions in mice (Figure 5A and B) and significantly lengthened the life span of mice intravenously injected with ACC-2^Ar^ cells by almost 5 days (Figure 5C and D). All above data revealed the enhanced metastatic abilities of the transformed cells that could be blocked by the EGFR inhibitor gefitinib, suggesting the potential preventive effects against ACC metastasis by targeting EGFR pathway.

The article "Epithelial Mesenchymal Transition Is Required for Acquisition of Anoikis Resistance and Metastatic Potential in Adenoid Cystic Carcinoma" was retracted in 2014. Reasons: errors in the cell lines or tissues; unreliable results or conclusions.

**Figure 5:** Prevention of ACC^Ar^ and EGF-induced metastasis *in vivo* by gefitinib. For *in vivo* metastasis analyses, the pulmonary metastatic models of mice were established by injected with ACC cells with indicated treatment by tail vein. The ACC-2 cells were pretreated with EGF (10 ng/ml) for 48 h, and gefitinib (1 µM) for 1 h, as well as ACC-2^Ar^ were used in the assays. ACC-2 parental cells were also injected as Control. A, Representative hematoxylin and eosin-stained histological sections of lungs from the mice injected with ACC cells. B, Quantitative analysis of pulmonary metastasis from mice as described above. Lesions of 0.1 mm or higher were counted from 20 slides per treatment (Mean ± SE, n = 5 for each group, *p<0.05 versus ACC-2). C, Survival curve of the mice with indicated treatments. The survival analysis were performed by OriginPro (n = 5 for each group, *p<0.05 versus ACC-2). D, Survival times of the mice as indicated treatments were expressed as Mean and SD.

### Slug-Mediated EMT-Like Transformation is Required for Anchorage-Independent Growth, Migration, and Invasion in ACC^Ar^ Cells

As EMT-like transformation was accompanied by the formation of anoikis resistance in both ACC^Ar^ and EGF-stimulated ACC cells, it was reasonable for us to investigate whether EMT was required for the acquisition of anoikis resistance in these cells. RNAi-mediated knockdown of Slug reversed EMT in these variant cells, manifesting as the morphological reversal of ACC-2^Ar^ to its cobblestone shape, compared with the NC group (Figure 6A and B). As the major epithelial marker, E-cadherin was observed to relocalize at the adherens junctions of the cells and restored protein expression levels (Figure 6A and B). Meanwhile, the expression of vimentin was significantly down-regulated after ACC^Ar^ and EGF-treated cells were infected with Slug siRNA (Figure 6A).

**Figure 6:** Requirement of Slug-mediated EMT in acquisition of anoikis resistance and migration/invasion. ACC-2^Ar^ and ACC-2 were transfected with Slug siRNA and NC siRNA. The ACC-2-transfected cells were then stimulated with EGF (10 ng/ml). A, The protein expression levels of Slug, E-cadherin, and vimentin were determined using Western blot analysis. B, The morphology and expression of E-cadherin were analyzed by immunofluorescence. C, Apoptosis in suspension was measured using Cell Death Detection ELISA^PLUS^ (Mean ± SE, **p<0.01 versus ACC-2^Ar^ with NC siRNA treatment). D, Anchorage-independent growth was analyzed using soft agar assay. Quantitative analyses were performed by counting the visible clones using ImageJ. The results were expressed as relative ratio to ACC-2 with pEGFP transfection (Mean ± SE, **p<0.05 versus ACC-2 with NC siRNA transfection, ##*p*<0.05 versus ACC-2^Ar^ with NC siRNA transfection). E, ACC-2 cells were transfected with NC siRNA and Slug siRNA, respectively, and then cultured in suspension. The EGFP protein was carried by the lentivirus as marker. The number of EGFP-positive cells was counted by flow cytometry and represented as relative ratio to ACC-2 cells cultured in adhesion (Mean ± SE, *p<0.05 versus ACC-2 in adhesion). F, Migration (top panel) and invasion (low panel) were determined using transwell Boyden systems coated without and with Matrigel, respectively.

The article "Epithelial Mesenchymal Transition Is Required for Acquisition of Anoikis Resistance and Metastatic Potential in Adenoid Cystic Carcinoma" was retracted in 2014. Reasons: errors in the cell lines or tissues; unreliable results or conclusions.

The apoptosis induced by detachment in variants and EGF-treated cells was analyzed using Cell Death Detection ELISA^PLUS^. As shown in Figure 6C, apoptosis evasion in ACC^Ar^ and EGF-treated cells was significantly blocked by Slug siRNA. Furthermore, the survivability of these cells in anchorage-independent conditions was measured using soft agar assay. The results indicated that depletion of Slug markedly suppressed the anchorage-independent growth of both ACC^Ar^ and EGF-treated cells (Figure 6D). In addition, to analyze the role of EMT in the formation process of anoikis resistance, we cultured ACC-2 cells infected with Slug or negative control (NC) siRNA (labeled with GFP as biomarker), as previously described with rounds of suspension and adhesion. The results revealed that GFP-positive cells under fluorescence microscope diminished with the culture rounds, indicating that these cells, which were unable to undergo EMT, were undergoing apoptosis in suspension (Figure 6E). Finally, the aggressive characteristics of ACC^Ar^ or EGF-treated cells were analyzed using migration and invasion assays performed in a transwell system. The results showed that knockdown of Slug significantly suppressed migration or invasion of these cells, confirming that EMT plays an essential role in the metastasis of ACC (Figure 6F). Taken together, all above results suggested that Slug-mediated EMT-like transformation was essential for the anoikis resistance of the variants, as well as enhanced migration and invasion.

The article "Epithelial Mesenchymal Transition Is Required for Acquisition of Anoikis Resistance and Metastatic Potential in Adenoid Cystic Carcinoma" was retracted in 2014. Reasons: errors in the cell lines or tissues; unreliable results or conclusions.

### Overexpression of Twist or Slug is Enough to Induce EMT and Acquisition of Anoikis Resistance

Having confirmed that Slug-mediated EMT is essential to anoikis resistance, migration, and invasion in ACC cells, we therefore investigated whether EMT induced by overexpression of Slug or Twist could generate anoikis-resistant abilities in ACC cells. Thus, we constructed and transfected overexpression plasmids of Twist and Slug into ACC-2 cells. After selecting the stable clones, we observed dramatic morphological changes compared with the controls (pEGFP) that were similar to the transformation in ACC^Ar^ cells (Figure 7A). Moreover, we detected up-regulation of vimentin and down-regulation of E-cadherin, indicating that EMT can be induced by the overexpression of Twist or Slug (Figure 7B). We then assessed the anoikis-resistant abilities in suspension and migration/invasion capabilities *in vitro* of these transformed cells. The results demonstrated that these clones were more fragile to detachment-induced apoptosis compared with the ACC^Ar^ cells but much blunter compared with parental ACC cells under such conditions (Figure 7C). Similar results were also found for anchorage-independent growth in soft agar assay (Figure 7D). Migration and invasion assays performed with a transwell Boyden system showed increased cell numbers across the semipermeable membrane compared with the parental ACC cells (Figure 7E). These results indicated that forced EMT in ACC cells by overexpression of EMT-related transcription factors contributed to the acquisition of anoikis resistance and migration/invasion although that its effects on anchorage-independent growth declined compared with ACC^Ar^ cells.

**Figure 7:** Prevention of apoptosis in ACC cells in suspension by EMT induction. The ACC-2 cells were transfected with pEGFP, pEGFP-Twist, and pEGFP-Slug. A, The morphology and location of E-cadherin were analyzed by immunofluorescence. B, The protein expression levels of Slug, Twist, E-cadherin, and vimentin were determined using Western blot analysis. C, Apoptosis in suspension was measured using Cell Death Detection ELISA^PLUS^ (Mean ± SE, *p<0.05 versus ACC-2 with pEGFP transfection, #*p*<0.05 versus pEGFP-Twist group). D, Anchorage-independent growth was analyzed using soft agar assay Quantitative analyses were performed by counting the visible clones using ImageJ. The results were expressed as relative ratio to ACC-2 with pEGFP transfection (Mean ± SE, **p<0.05 versus ACC-2 with pEGFP transfection, ##*p*<0.05 versus pEGFP-Twist group). E, Migration and invasion were determined using transwell Boyden systems coated without and with Matrigel, respectively. F, The mRNA expression levels of VEGF, MMP9, and SDF-1α were analyzed using qRT-PCR, and the results were expressed as relative ratio to ACC-2 transfected with pEGFP (*p<0.05 versus ACC-2 pEGFP group, **p<0.01 versus ACC-2 pEGFP group).

The article "Epithelial Mesenchymal Transition Is Required for Acquisition of Anoikis Resistance and Metastatic Potential in Adenoid Cystic Carcinoma" was retracted in 2014. Reasons: errors in the cell lines or tissues; unreliable results or conclusions.

### Expression of EMT-Related Genes in ACC and its Correlation with EGFR Activation

To make our present work more clinically significant, we investigated the natural status of EGFR, as well as the expression levels of EMT-related genes in ACC tissues. Representative immunohistochemical results for the selected cases are shown in Figure 8A. EGFR was moderately stained in the cytoplasm of most ACC cells, especially in the solid type, which is considered to be the most aggressive of the three pathological types of ACC. We next identified the expression levels of EMT-related genes in ACC tissues via serial sections. Membranous or cytoplasmic staining of E-cadherin in ACC was much lower than that in normal salivary glands, and even lost in some cases. In addition, Slug was strongly stained in the nucleus of tumor cells in ACC, suggesting that EMT frequently occurs in ACC. Serial section immunohistochemistry revealed that loss of E-cadherin was generally linked with the expression of Slug, and Spearman’s rank test showed that E-cadherin staining and Slug were negative correlated (*p* = 0.0263, Figure 8B). The significant correlation between EGFR and Slug was confirmed using Spearman’s rank test (*p* = 0.0481, Figure 8B). MMP9, as a marker of metastasis or invasion, was also analyzed. The results from serial sections showed that intensive staining of MMP9 in the cytoplasm was consistent with the positive staining of EGFR. All these results indicate that EMT, manifesting as loss of E-cadherin and nuclear expression of Slug, is significantly correlated with the positive staining of EGFR, which potentially helps promote metastasis in ACC.

**Figure 8:** Expression levels of EGFR, Slug, E-cadherin, and MMP9 in ACC tissues. A, Representative immunohistochemical staining of EGFR, Slug, E-cadherin, and MMP9 in human adenoid cystic carcinoma and negative gland tissue (NSG). B, Spearman’s correlation were used to determine the relationship between EGFR and Slug (left panel) and that between Slug and E-cadherin (right panel) (*p*<0.05). Histoscore based on quantification as described in the method and statistics with OriginPro.

## Discussion

In this study, we investigated the role of EMT-like transformation in the acquisition of anoikis resistance in ACC cells and determined the therapeutic effects of targeting the EGFR/PI3K/Akt signaling pathway in the metastasis of human ACC.

The article "Epithelial Mesenchymal Transition Is Required for Acquisition of Anoikis Resistance and Metastatic Potential in Adenoid Cystic Carcinoma" was retracted in 2014. Reasons: errors in the cell lines or tissues; unreliable results or conclusions.

Metastasis of human ACC is a major cause of mortality [2]. The prognosis for patients with ACC depends mainly on the control of distant metastasis rather than on the success of locoregional cure [25]. Metastasis is a complex multistep process that includes local invasion, intravasation, survival in the circulation, arrest in capillaries, extravasation, and, finally, outgrowth to produce macrometastasis to distant organs [5], [26]. Resistance against anoikis is considered a prerequisite for cancer cells to survive in the circulation [8]. The present study detected an EMT-like transformation in ACC^Ar^ cells, in accordance with previous studies showing that most tumor cells in the circulation, usually termed circulating tumor cells (CTCs), lost their epithelial markers and underwent EMT-like transformation [27]. Thus, the method for detection and isolation of CTCs in patients based on the capture of epithelial cell adhesion molecules [28] should be modified according to our study. Generally, EMT is described as a process that endows cancer cells with motility to shed from primary sites and intravasate into the circulation [7]. The present study confirmed that EMT-like transformation also contributed to the survival of tumor cells in the circulation, highlighting the complex and multiple roles of EMT in cancer metastasis. Although several studies have shown that there are more CTCs in the circulation of patients with cancer [29], [30], the incidence of metastasis is quite small. The results from our study suggest that only those transformed cells can survive in the circulation and finally form micrometastases to distant organs.

The transcription factors that repress the expression of E-cadherin, such as Twist, Snail, and Zeb1, among others, have been described as central mediators in EMT-like transformation [31], [32]. In our experiments, Slug proved to be a crucial transcription factor in EMT-like transformation. Distinct from other EMT-related transcription factors, Slug is considered to contribute to the function of stem cells via the c-kit signaling pathway or by suppressing p53 transcriptional activities [33]–[35]. A recent study reported that Slug and Sox9 were sufficient to convert differentiated luminal cells into stem cells and contributed to the tumorigenic and metastasis-seeding abilities of human breast cancer cells, suggesting that Slug has a more important role in cancer progression [36]. Moreover, our unpublished data also showed that the expression of CD44, a marker of cancer stem cells, was increased in these anoikis-resistant variants and that overexpression of Slug in ACC cells was sufficient to up-regulate the expression of this molecule. To confirm the essential role of Slug in EMT-like transformation and the acquisition of anoikis resistance in ACC cells, we suppressed Slug expression using RNAi. Down-regulation of Slug significantly increased the apoptosis rate of variant cells in suspension, reduced growth in anchorage-independent conditions, and reversed the EMT-like transformation, indicating that Slug-mediated transformation is required for the acquisition of anoikis resistance in ACC cells. Moreover, by blockade of Slug elevation in parental ACC cells, we succeeded in alleviating the formation of anoikis resistance in parental ACC cells. Moreover, we investigated whether induction of EMT by forced overexpression of Slug or Twist could rescue the cells from death in suspension. Overexpression of Slug or Twist was sufficient to induce EMT-like transformation, enhanced the migration and invasion abilities of ACC cells, and contributed to anoikis resistance in ACC cells, albeit only partially, suggesting that other survival pathways are involved in anoikis resistance in these variant cells.

The article "Epithelial Mesenchymal Transition Is Required for Acquisition of Anoikis Resistance and Metastatic Potential in Adenoid Cystic Carcinoma" was retracted in 2014. Reasons: errors in the cell lines or tissues; unreliable results or conclusions.

Previous studies have demonstrated in many cases that growth factor signaling pathways mediating the EMT process might also contribute to anoikis resistance [37], [38]. In the present study, we proved that the EGFR/PI3K/Akt signaling pathway acts as the common regulator for EMT-like transformation and the acquisition of anoikis resistance in ACC cells. qPCR and Western blot analysis confirmed the elevation of EGF, and the phosphorylation of EGFR notably increased in ACC^Ar^ cells compared with their parental cells, indicating the probable role of EGF/EGFR in variant ACC cells. Thus, we stimulated ACC cells with EGF and found that EGF was sufficient to induce EMT-like transformation and prevent tumor cells from detachment-induced apoptosis. To uncover the underlying mechanism through which EGF induces such processes, we investigated the probable pathways previously reported as the downstreams of EGFR. As numerous studies have shown that the activation of EGFR promotes cancer invasion and metastasis in a PI3K/Akt- and/or MEK/ERK-dependent manner [10], [21], [39], [40], we measured the activation of Akt and ERK in our experiments. We found that phosphorylation of PI3K, p85, and Akt was significantly increased in detachment-selected and EGF-treated cells and that the phosphorylation level of ERK did not significantly change in both conditions. Furthermore, pretreatment with the PI3K-specific inhibitor LY294002 completely reversed the EMT-like transformation induced by EGF or anoikis-resistant variant cells via the down-regulation of Slug and alleviated the survivability of these cells in suspension. According to these findings, we hypothesized that the therapeutic mechanism against EGFR activation is a promising means of preventing metastasis of human ACC. Therefore, we selected gefitinib, a highly selective, reversible inhibitor of the tyrosine kinase domain associated with EGFR that has demonstrated efficacy in patients harboring EGFR overexpression or mutations [41]–[43], for our experiments. Having confirmed the solid effects of this pharmacological inhibitor on the reversal of EMT-like formation and suppression in anoikis via *in vitro* studies, we therefore established a nude mouse model of pulmonary metastasis to examine its therapeutic effects on the metastasis of ACC cells *in vivo*. The results showed that pretreatment with gefitinib significantly decreased the pulmonary metastatic formation abilities of the anoikis-resistant variant cells and promoted survival of the mice. All these findings strongly suggest that targeting EGFR/PI3K/Akt holds promising therapeutic efficacy in human ACC.

The article "Epithelial Mesenchymal Transition Is Required for Acquisition of Anoikis Resistance and Metastatic Potential in Adenoid Cystic Carcinoma" was retracted in 2014. Reasons: errors in the cell lines or tissues; unreliable results or conclusions.

To make the above-mentioned findings more clinically significant and therapeutically meaningful, we then investigated the natural expression status of EGFR signaling and the EMT inducer Slug in ACC specimens. Previous studies have reported that EMT-related genes, such as Snail, Twist, and Sip1, are frequently observed in cases of human ACC [44], [45] and proved to be associated with poor outcomes and high metastasis rates in patients [44], [46], [47]. Our results showed that EGFR overexpression is correlated with the expression of Slug, indicating that aberrant activation of EGFR signaling induces EMT and further promotes tumor metastasis. In addition, we investigated E-cadherin and vimentin to validate whether EMT occurred in the patients with ACC. Our immunohistochemical staining results revealed that loss of E-cadherin and acquisition of vimentin frequently occurred in ACC specimens, especially in cells adjacent to the stroma, suggesting that the interaction between cancer cells and mesenchymal cells may contribute to these processes.

In conclusion, this study has confirmed that induction of EMT-like transformation is required for the acquisition of anoikis resistance in ACC cells. Our research has also revealed that activation of the EGFR/PI3K/Akt signaling pathway is responsible for both EMT-like transformation and anoikis resistance in ACC, pointing to the potential therapeutic value of targeting such pathways in preventing distant metastasis of human ACC.

## Supporting Information

Figure S1 **Anoikis resistant variants of ACC cells showed alleviated proliferation compared to parental cells.** MTT assays were performed to measure the proliferation rate of ACC cells.
(TIF)

Figure S2 **The mRNA expression of epithelial and mesenchymal markers in anoikis resistant variants of ACC cells.**
(TIF)

Figure S3 **Confirmation of the efficacy of RNA interference against Slug.**
(TIF)

Protocol S1 (DOC)
